# Effect of Maternal Triclosan Exposure on Neonatal Thyroid-Stimulating Hormone Levels: A Cross-Sectional Study

**DOI:** 10.1155/2022/3082304

**Published:** 2022-09-28

**Authors:** Elham Attarian, Karim Ebrahimpour, Mohammadreza Maracy, Seyede Shahrbanoo Daniali, Bahareh Shoshtari-Yeganeh, Malihe Moazeni, Afshin Ebrahimi, Roya Kelishadi

**Affiliations:** ^1^Student Research Committee, School of Health, Isfahan University of Medical Sciences, Isfahan, Iran; ^2^Department of Environmental Health Engineering, School of Health, Isfahan University of Medical Sciences, Isfahan, Iran; ^3^Environment Research Center, Research Institute for Primordial Prevention of Non-Communicable Disease, Isfahan University of Medical Sciences, Isfahan, Iran; ^4^Department of Epidemiology and Biostatistics, School of Health, Isfahan University of Medical Sciences, Isfahan 81676-36954, Iran; ^5^Department of Pediatrics, Child Growth and Development Research Center, Research Institute for Primordial Prevention of Non-Communicable Disease, Isfahan University of Medical Sciences, Isfahan, Iran

## Abstract

**Objective:**

This study is aimed at assessing the relationship between maternal urinary triclosan (uTCS) exposure and the thyroid-stimulating hormone (TSH) level of infant cord blood.

**Methods:**

This cross-sectional study was carried out in 2019-2020 in Isfahan, Iran, and 99 pregnant women participated in the study. Urine samples were collected after the 28th week of pregnancy, and the concentration of TCS was measured using GC/MS. The cord blood levels of TSH (CBL-TSH) were measured. The association between uTCS and CBL-TSH was examined based on the general linear model.

**Results:**

TCS was detected (≥0.01 ng/mL) in 100% of the urine samples, with the interquartile range (25%-75%) of uTCS levels 0.6-6.23 *μ*g/g Cr. uTCS was not associated with CBL-TSH after adjustment for covariates. A significant relationship was observed between CBL-TSH of neonates born to mothers who had given birth only once compared to mothers who had given birth twice or more times.

**Conclusions:**

Maternal exposure to TCS did not affect the infant CBL-TSH. However, the high concentrations of TCS in maternal urinary samples indicate the necessity of more precise regulations to decrease the use of this chemical in the industry and increase public awareness about using TCS-free compounds.

## 1. Introduction

Triclosan (TCS) or 5-chloro-2-(2,4-dichlorophenoxy)phenol is a synthetic lipid-soluble and broad-spectrum antimicrobial compound [1] which widely used in personal care products, daily household chemicals, and health products [2]. It is utilized in consumer products, including soaps, toothpaste, shampoos, mouthwashes, kitchenware, textiles, cleaning products, and personal care products such as cosmetics [3]. Typically, its concentration in personal care products is about 0.1-0.3% of product weight [4]. Human exposure to TCS usually occurs when consuming the products mentioned above, through dermal absorption, or exposure to other environmental factors, e.g., indoor and outdoor polluted air [3]. The estimated biological half-life of TCS is 21 hours, so it can be detected in urine, plasma, and breast milk in the human body that absorbs TCS mainly through the mouth and skin [5, 6]. TCS is also detected in cord blood and amniotic fluid [7]. TCS in the maternal serum of pregnant women can pass the placental barrier and arrive at the fetus; thus, it can be detected in neonatal cord blood [8].

The chemical structure of TCS is similar to estrogenic and androgenic endocrine disruptor chemicals (EDCs) such as polychlorinated biphenyls (PCBs), polybrominated diphenyl ethers (PBDEs), bisphenol A, and dioxins [4]. Some studies showed that TCS, as an essential EDC, can affect estrogen, testosterone, and thyroid hormone levels [9]. TCS may alter thyroid homeostasis, which is especially significant for pregnant women due to the need for thyroid hormones in their normal reproduction [10]. Some human studies reported that uTCS concentration increases during pregnancy or childbirth, and it might thus decrease maternal or neonatal thyroid hormone concentrations [11]. In turn, it may reduce thyroxine levels during pregnancy with adverse effects on fetal growth and neurodevelopment [12]. An in vivo study showed a decrease in the serum of total T4 and T3 hormones in a dose-response procedure in mice following exposure to TCS, as well as a reduction in total T4 in pregnant mice [13].

Because pregnant women and their fetuses are vulnerable to endocrine disorders, understanding the exposure to particular contaminants such as TCS and their consequences in pregnant women is of particular importance. Thus, it is critical to study the pregnant women population given their sensitivity to environmental chemicals such as TCS. Therefore, this study is aimed at assessing the relationship between the maternal urinary concentration of TCS and CBL-TSH. This is the first study in Iran to examine the relationship between the concentration of uTCS in pregnant women and TSH in their infant umbilical cord as sensitive and vulnerable groups.

## 2. Materials and Methods

### 2.1. Study Population

This cross-sectional study approved by the Ethics Committee of Isfahan University of Medical Sciences was carried out in 2019-2020 as a substudy of the prospective epidemiological research studies in Iran (PERSIAN) birth cohort entitled “Isfahan Birth Cohort” (IBC). All participants signed informed consent for participation in the study. Detailed information about the study design, participants, and data collection method can be found in a previously published article [14]. However, in summary, the primary cohort has more than 3000 participants. A total of 99 pregnant women participated in the study to investigate the relationship between maternal uTCS concentrations and their infant's CBL-TSH.

### 2.2. Inclusion Criteria

Inclusion criteria are as follows: the participants (1) whose delivery was not emergency, (2) were randomly selected (based on a table of random numbers), (3) were informed about the objectives and protocols of the study and follow-up stages, (4) filled in the questionnaires, (5) had spot urinary and cord blood samples taken, (6) were reassured that their information would be kept confidential, (7) had been living in Isfahan for at least in last year, (8) were in the third trimester, and (9) intended to give birth in Isfahan hospitals.

### 2.3. Exclusion Criteria

In this study, the exclusion criteria were chosen as Wang et al.'s study with some modifications. All participants with (a) a failure to provide a urine sample, (b) a history of smoking and alcohol consumption before and during pregnancy, and (c) having urine samples with creatinine levels ≤ 0.05 g/L and ≥3 g/L were excluded from the study [8]. It should be noted that in our selected samples in this study, no sample included the exclusion criteria. Therefore, 99 samples were surveyed and examined.

### 2.4. Studied Variables

The data obtained from various questionnaires completed in the cohort designed by mothers in the third trimester were surveyed. These data include eating habits, body mass index (BMI), physical activity, age of mother, number of deliveries, supplementation use during pregnancy, gestational diseases (diabetes, thyroid, and hypertension), and environmental exposures (cosmetic use). Moreover, the infants' sexes were extracted from the completed questionnaires.

### 2.5. Collection of Urine Samples

First, 20 mL of pure morning urine was taken from each subject in the third trimester of pregnancy and collected in polyethylene containers. After, they were transferred to the laboratory and reserved at -70°C until analysis. In addition, to determine the creatinine levels, 5 mL of the sample was taken, and the rest was used to determine the TCS content.

### 2.6. Measurement of uTCS Concentration

All solvents, standards, and derivatives, including 1,1,1-trichloroethane, methanol, N-(tert-butyldimethylsilyl)-N-methyltrifluoroacetamide (MTBSTFA) derivative compounds, and TCS standards, were purchased from Sigma-Aldrich Co., USA. To measure the concentration of TCS in urine, the dispersed liquid-liquid microextraction (DLLME) method was employed, followed by gas chromatography equipped with a mass spectrometry detector (GC/MS) [15]. Briefly, urine samples were liquefied at room temperature, and then, a specific volume of the sample was taken and diluted to 5 mL with distilled water. Next, a mixture of two solvents of methanol (750 *μ*L as the dispersant solvent) and trichloroethane (60 *μ*L as the extracting solvent) was suddenly added to the sample, and it was centrifuged at 5000 rpm for 5 min. The extracted solution was transferred to a microtube with a syringe and then dried with N_2_ gas. Subsequently, 20 *μ*L of the MTBSTFA derivative compound was added to the microtube and was mixed vigorously by a vortex, and the microtube was then placed in a water bath for 1 min at 60°C. Finally, 2 *μ*L of the solution was injected into the GC/MS device (Model A7890, Agilent Technology, USA) to determine the TCS concentration. The GC/MS apparatus had a 30 m long DM5-MS capillary column, a diameter of 0.25 mm, and an internal film thickness of 250 *μ*m. The injector temperature was set at 280°C with a split ratio of 5 : 1, and the injection volume was 2 *μ*L. The carrier gas flow rate was set at 1 mL/min. The initial oven temperature was 80°C for 1 min, which was increased to 270°C at 10°C per minute. A total run time of 22 min was obtained for each injection. To minimize dilution differences between urine samples, TCS concentrations were adjusted by creatinine levels. For this purpose, the levels of creatinine in the urine samples were determined by the Jaffe-kinetic method and an Alpha Classic-AT device in Isfahan University Jihad Medical Diagnostic Laboratory, and the concentration of TCS was expressed relative to creatinine.

### 2.7. Measurement of TSH Levels

The cord bloods were collected after the infants were delivered, and the umbilical cord was cut. The sampling was done by a trained midwife separating the infant from the placenta, immediately after clamping of the two sides of cord blood before the natural clotting process begins. After cleaning the cord with alcohol, 4 mL blood was collected from the vein and stored in an EDTA tube, mixed by inverting 4-5 times, and then transmitted to a reputable laboratory [16]. The collected neonatal cord blood serum samples were stored at -40°C until the TSH assay. TSH levels were determined by the chemiluminescence immunoassay (CLIA) method using the Liaison Hormone Tester [17]. This measurement was performed in Milad Medical Diagnostic Laboratory of Isfahan.

### 2.8. Quality Assurance/Quality Control (QA/QC)

According to ICH guidelines, all GC/MS methods should be approved for precision, accuracy, and linearity [18]. The samples' standard deviations (SD) were calculated and used for precision assessment of the analysis in triplicate and reported as intra- and extraday RSDs% (relative standard deviation). In addition, the HPLC grade water was used as a blank sample in triplicate instead of human urine for the assay method accuracy evaluation. The detection limit (LOD) and limit of quantification (LOQ) values of the analyses, considered in terms of signal to noise, were calculated to be 3 and 10, respectively.  Table 1 shows the validation procedure results and QA/QC parameters of the method.

### 2.9. Statistical Analysis

Qualitative data are expressed as frequency (percentage) and quantitative as mean ± SD. The statistical analysis results showed that TCS and TSH did not have a normal distribution. The GLM regression model with a gamma link was used to assess the relationship between the measured TCS concentration, TSH levels, and other variables, including lifestyle variables (physical activity, eating habits, and BMI), pregnancy variables (number of deliveries, infant sex, supplementation use during pregnancy, gestational diseases of the thyroid, diabetes, and blood pressure), age of mother, and environmental exposure to cosmetics. SPSS 20 (SPSS, Chicago, IL, Inc.) was used for all statistical analyzes.

## 3. Results

The characteristics of mothers and their infants are presented in Table 2. The mean and SD of maternal BMI during pregnancy was 28.65 ± 4.34 kg/m^2^. The pregnant women used cosmetics and personal care products by 69.7% (*n* = 69) and 60.6% (*n* = 60), respectively. The results showed that 85 participants (86%) had low physical activity, and only about 14 participants (14.1%) had moderate-to-severe physical activity. Furthermore, 38 pregnant women (38.4%) had <2 deliveries, while 61 (61.6%) had >2. In terms of pregnancy disease, 11 mothers (11.1%) had hypothyroidism, and 8 (8.1%) had diabetes.

Table 3 lists the maternal uTCS concentrations and CBL-TSH. TCS was detected in 100% of the urine samples (*n* = 99). The mean ± SD concentrations of TCS relative to creatinine and TSH were 4.81 ± 6.11 *μ*g/g Cr and 8.96 ± 7.41 MIU/L, respectively.

The relationship between CBL-TSH, uTCS concentration, and other variables was evaluated using the GLM regression model with gamma link (Table 4). There was no significant relationship between the concentration of TCS in urine samples and the level of TSH in the neonatal umbilical cord (*P* value = 0.962). Moreover, there was a difference in the level of TSH in the umbilical cord of neonates born to mothers who had given birth only once (*P* value = 0.014) compared to mothers who had given birth two or more times (*P* value = 0.480). In other words, neonates born to mothers who had given birth only once had higher CBL-TSH.

## 4. Discussion

This study surveyed the possible association between the uTCS concentration of mothers and CBL-TSH. There was no significant correlation between increased maternal uTCS concentration and increase/decreased neonatal CBL-TSH (*P* value = 0.962). Therefore, few studies have examined the relationship between maternal uTCS concentration and CBL-TSH. The results of some of these are in accordance with the findings of this research. Wang et al. stated that there was no significant relationship between maternal uTCS concentration and cord blood FT4 or TSH concentration. They also presented a negative association between maternal uTCS and FT3 levels in cord blood [8]. Berger et al. also found no association between TCS concentrations and neonatal thyroid-stimulating hormones [19]. The results of Braun et al.'s study indicated that the average concentration of pregnancy uTCS was negative associated with TT4 and FT3 concentration in cord blood, while it was positive associated with CBL-TSH [20].

The difference between our study and most other studies is that they examined other hormones, including T3 and T4, in mothers' serum and in the neonatal umbilical cord instead of TSH. Based on the results of the present study and others, TCS does not affect infants' CBL-TSH. However, some studies demonstrated the effect of TCS on reducing or increasing T3 and T4 hormones in infants' umbilical cords [8]. EDCs are a diverse group of chemicals involved in raising and inhibiting hormone signaling [21]. It has been suggested that the placenta is a target organ that exposes to organic compounds like TCS during pregnancy [22].

In the present study, there was no association between infant sex and a decrease or increase in TSH concentration (*P* value = 0.312). Furthermore, many previous studies said no significant difference between the CBL-TSH and the neonates' sex [17, 23, 24]. On the contrary, some studies reported that male neonates have higher TSH concentrations than female neonates [25–27].

In this study, it was not found a significant relationship between BMI and maternal age during pregnancy and TSH concentration (*P* value > 0.05). In addition, other studies showed that BMI and maternal weight gain was not associated with CBL-TSH [23, 25]. However, the survey by Kahr et al. reported a relationship between maternal obesity with increased cord TSH concentrations. Still, it should be noted that this association may only apply at the extremes of maternal weight [28].

Generally, the activation of estrogen receptors can affect insulin resistance and glucose metabolism [29]. Babies of diabetic mothers have a lot of metabolic abnormalities, like those observed in premature infants. That thyroid hormone might have a role in the resistance of these metabolic pathways. In premature infants, thyroid function decreased compared with normal newborns in the first days of life [30]. In this regard, numerous studies have found that TCS has estrogenic properties and effects on the endocrine [31]. In the present research, no significant relationship was observed between CBL-TSH and gestational diseases such as diabetes (*P* value = 0.277) and hypothyroidism (*P* value = 0.446). In addition, in previous studies, there was no significant correlation between CBL-TSH with hypothyroidism and gestational diabetes [25, 26]. Furthermore, several studies did not find any important relationship between maternal diabetes and CBL-TSH [23, 25, 30]. In contrast, a study that evaluated gestational diabetes reported the relationship between gestational diabetes with higher TSH levels in cord blood. However, this increase may be a function of stress increasing in infants of mothers with gestational diabetes mellitus [32].

As previously stated, in the present study, a significant relationship between mothers who had a single delivery (*P* value = 0.014) in comparison with mothers who had more than one (*P* value =0.480) with the concentration of TSH in the umbilical cord was found. In other words, mothers who gave birth once had higher levels of TSH in their fetal umbilical cord than mothers who gave birth twice or more. Similar to the findings of our study, several studies have reported an increase in the cord TSH level in first-born neonates compared to later-born ones [26, 27, 33]. Moreover, some studies have reported that first infants have higher TSH concentrations than subsequent ones [26, 30, 34]. In contrast, one study from Belgium reported no differences in TSH levels according to birth order [24]. This might be as a result of a confounding factor about environmental exposures such as some persistent chemicals that are present in higher levels in first-born children than in subsequent births [25].

Cosmetic and healthcare products are important sources of human exposure to TCS [3]. TCS has been identified in 16 cosmetics, constituting about 10% of all products [35]. This compound is an antimicrobial agent in cosmetic and personal care products to prevent or reduce bacterial and fungal infections. It is easily absorbed into the skin, and exposure to it can lead to hormonal and reproductive disorders and affect the immune response [36]. Based on our results, no correlation was found between mothers' use of cosmetics during pregnancy and CBL-TSH (*P* value = 0.7). TCS has been popular in the food packaging industry owing to its antimicrobial properties and is used in plastic materials to ensure the durability and safety of products. Because TCS can be released from the surface of materials used in packaging of food, it was removed from the EU list in March 2012 for use in food contact plastics [4]. The results of our research also indicated that the lack of use of plastic containers for storing water was not associated with TSH concentrations in cord blood (*P* value = 0.083).

Table 5 presents the uTCS concentration in pregnant women and infant CBL-TSH reported in different studies. The results of the current study were in line with others regarding TCS concentrations in urinary samples of pregnant women. Furthermore, the geometric mean concentration of TCS in this study was 0.45 *μ*g/g Cr, which is lower than the other studies [8, 37]. The geometric mean TSH concentration was 1.94 MIU/L, which shows a lower value than that reported by Wang et al. in 2017 (1.5 MIU/L) [8].

### 4.1. The Limitations of the Study

The main limitation of the current study was its cross-sectional design, which could not show the long-term effects of triclosan exposure on the health of mothers and infants from different aspects. Using spot urine samples, which may not reflect prolonged exposure, is another limitation of the present study. In addition to TSH, the association of TCS with other hormones such as T3 and T4 should be investigated, and a larger sample should be recruited to investigate this association. Significant limitations of such studies are participants' lack of cooperation with the research team and the time and costs of tests. We did not examine other potential factors related to the TSH level, e.g., thyroid antibodies, markers of inflammation, and genetic factors. However, our study was one of the first studies and can provide information for future studies with more sophisticated laboratory tests.

## 5. Conclusions

In the present study, there was no significant association between maternal uTCS and CBL-TSH at the third trimester of pregnancy. Although maternal exposure to TCS may not affect infant CBL-TSH, given that these results are according to cross-sectional data, the results should be interpreted with caution. The significant concentration of TCS observed here necessitates more precise regulations in the industry to limit the use of this substance in products and the importance of public education for women of childbearing age to use alternative products that are TCS-free.

## Figures and Tables

**Table 1:** The parameters of QA/QC for TCS determination.

R^2^^∗^	Precision (%RSD)		LOD^∗∗^ (*μ*g/L)	LOQ^∗∗∗^ (*μ*g/L)	Recovery (% ± SD)
	Within a day	Outside a day			
0.995	4.3	5.3	0.04	0.11	100±6.5

^∗^ *R*-squared correlation. ^∗∗^Limit of detection. ^∗∗∗^Limit of quantitation.

**Table 2:** Characteristics of mothers and their infants.

Characteristic	Categories	n (%)/Mean ± SD
Maternal		
Pregnancy BMI (kg/m^2^)		28.65±4.34
Age (years)	19-29	55(55.6)
	30-40	39(39.4)
	>40	5(5.1)
Cosmetic usage	Yes	69(69.7)
	No	30(30.3)
Personal care product∗	Yes	60(60.6)
	No	39(39.4)
Plastic packaging usage Water	Yes	24(24.2)
	No	75(75.8)
Physical activity	Low	85(85.9)
	Moderate to severe	14(14.1)
Number of deliveries	First	38(38.4)
	Second	38(38.4)
	Third or more	23(23.2)
Hypothyroidism	Yes	11(11.1)
	No	88(88.9)
Diabetes	Yes	8(8.1)
	No	91(91.9)
Infants		
Sex	Male	58(58.6)
	Female	40(40.4)

∗Including cream, lotion, ointment, oil, and powder. Among the variables studied in the study, including the use of supplements during pregnancy, since all participants in the study had used supplements, its relationship has not been examined and is not presented in the table. In addition, due to the involvement of only one person in the study of hypertension, this variable was not studied.

**Table 3:** Concentrations of TCS in maternal urine and TSH in cord blood of participants.

Concentration	*N*	Mean ± SD^∗^	Median (IQR)^∗∗^	Min-max
Maternal urine TCS measures				
TCS (ng/mL)	99	4.29 ± 5.16	2.89 (0.47-5.92)	0.02-30.39
Creatinine (g/L)	99	0.97 ± 0.52	0.88 (0.55-1.25)	0.18-2.7
Creatinine-adjusted TCS (*μ*g/g Cr)	99	4.81 ± 6.11	3.14 (0.6-6.23)	0.01-41.32
CBL-TSH (MIU/L)	98	8.96 ± 7.41	6.95 (4.2-10.42)	1.7-50.3

^∗^Standard deviation. ^∗∗^Interquartile range.

**Table 4:** The association of maternal TCS concentration and other studied variables with umbilical cord TSH hormone concentration using GLM model with gamma link.

Variables	Categories	TSH	
		*β*-Coefficient (95% CI)	*P* value
TCS (*μ*g/g Cr)		0.000 (-0.021-0.023)	0.962
Pregnancy BMI (kg/m^2^)		0.000 (-0.030-0.031)	0.990
All age groups (years)		0.093 (-0.155-0.344)	0.501
Plastic packaging (water)	Yes	—	—
	No	-0.296 (-0.608-0.005)	0.083
Physical activity	Low	-0.176 (-0.601-0.230)	0.525
	Moderate to severe	—	—
Number of deliveries	First	0.427 (0.019-0.828)	0.014
	Secondary	0.127 (-0.213-0.459)	0.480
	Third or more	—	—
Sex of infant	Male	—	—
	Female	-0.136 (-0.418-0.149)	0.312
Hypothyroidism	Yes	-0.111 (-0.515-0.330)	0.446
	No	—	—
Diabetes	Yes	-0.247 (-0.709-0.262)	0.277
	No	—	—
Cosmetic usage	Yes	0.054 (-0.256-0.36)	0.7
	No	—	—
Personal care product	Yes	0.169 (-0.119-0.452)	0.231
	No	—	—

**Table 5:** Urinary TCS concentration in pregnant women and baby umbilical cord TSH reported in different studies.

Concentration	Units	GM (95% CI)	References
TCS	*μ*g/g Cr	0.45	This study
TSH	MIU/L	1.94	
TCS	*μ*g/g Cr	6.00 (5.16, 6.96)	[8]
TSH	MIU/L	5.49 (5.21, 5.75)	
TCS	*μ*g/g Cr	0.81	[37]

## Data Availability

The data used to support the findings of this study are available in the manuscript.
